# Cases of replacing diffractive bifocal intraocular lens with extended depth of focus intraocular lens due to waxy vision

**DOI:** 10.1371/journal.pone.0259470

**Published:** 2021-10-29

**Authors:** Ryu Takabatake, Makiko Takahashi, Takuya Yoshimoto, Fumiaki Higashijima, Yuka Kobayashi, Chiemi Yamashiro, Kazuhiro Kimura

**Affiliations:** 1 Takabatake West Eye Clinic, Okayama City, Okayama, Japan; 2 Department of Ophthalmology, Yamaguchi University Graduate School of Medicine, Ube City, Yamaguchi, Japan; University of Toronto, CANADA

## Abstract

**Purpose:**

To investigate the postoperative course of patients who explanted a diffractive bifocal intraocular lens (IOL) due to waxy vision and implanted with an extended depth of focus IOL.

**Methods:**

This study evaluated 29 eyes of 25 patients who underwent diffractive bifocal IOL explantation followed by TECNIS Symfony^®^ implantation because of dissatisfaction due to waxy vision at the Takabatake West Eye Clinic between January 2018 and November 2019. The indication criteria for this surgery were patients with uncorrected distance visual acuity of 0.05 logMAR or better, without eye diseases that may affect visual function, and no dissatisfactions about photic phenomena. We investigated patient demographics, uncorrected and corrected visual acuity, manifest refraction, contrast sensitivity, subjective symptoms, time to IOL explantation, explanted IOL type, and spectacle independence.

**Results:**

The time to the IOL exchange after the initial IOL implantation was 55.3 ± 50.4 days (range: 14–196 days). The logMAR corrected distance visual acuity before and after IOL exchange were −0.13 ± 0.06 and −0.14 ± 0.06, respectively (p = 0.273). After IOL exchange surgery, the area under log contrast sensitivity function increased significantly from 1.07 ± 0.12 to 1.21 ± 0.12 (p < 0.001), and the waxy vision symptoms improved. The spectacle independence rate at the last visit was 88.0%.

**Conclusion:**

For patients who complain of waxy vision despite good visual acuity after diffractive bifocal IOL implantation, exchange to extended depth of focus IOL was considered one of the useful surgical options.

## Introduction

In recent years, patients have higher expectations from cataract surgery, and many patients desire independence from spectacles as a surgical outcome. After multifocal intraocular lens (IOL) implantation, good distance and near visual acuities can be obtained, and so high patient satisfaction is achieved by reducing dependence on spectacles and improving quality of life [1, 2]. While the expectations of patients are increasing, some patients complain about postoperative visual function, and it may be difficult to deal with them. The most common cause of dissatisfaction was waxy vision due to decreased contrast sensitivity [3, 4], and for cases without factors, such as refractive error and posterior capsule opacity, exchange to monofocal IOL is considered a useful treatment option [4–7]. However, being forced to wear spectacles after surgery can lead to further dissatisfaction.

Diffractive bifocal IOLs distribute incident light into distant and near images and lead to concerns that the contrast sensitivity will decrease due to light loss [1, 8–10]. A new type of presbyopia-correcting IOLs called the extended depth of focus IOLs (EDOF IOLs) were developed with the aim of reducing these side effects. These IOLs extend the depth of focus to increase the range of clear vision and provide natural appearance for patients without a decline of vision at intermediate distances. TECNIS Symfony^Ⓡ^ (Johnson & Johnson Surgical Vision, Santa Ana, California, USA) an EDOF IOL which maintains contrast sensitivity close to that of monofocal IOLs by suppressing light loss and correcting chromatic aberration using a unique diffraction technology [10, 11]. Since the structure and optical characteristics of EDOF IOLs are different from those of diffractive bifocal IOLs, waxy vision may be less likely to occur.

This study aimed to investigate the postoperative course of patients who had their diffractive bifocal IOLs explanted due to waxy vision and underwent EDOF IOL implantation.

## Patients and methods

### Patients

This retrospective study was approved by the institutional review board of Yamaguchi University and adheres to the tenets of the Declaration of Helsinki. All participants actively agreed to participate in the study and were given the choice to opt-out, in case they wished to. This study evaluated 29 eyes of 25 patients who underwent diffractive bifocal IOL explantation followed by TECNIS Symfony^®^ (including toric type) implantation because of dissatisfaction to waxy vision at the Takabatake West Eye Clinic between January 2018 and November 2019. The indication criteria for this surgery were as follows: (1) uncorrected distance visual acuity (UDVA) of 0.05 logMAR or better, (2) area under the log contrast sensitivity function (AULCSF) of 0.80 or better, (3) absence of eye diseases that may affect visual function, and (4) no dissatisfactions regarding photic phenomena (glare, halos, starburst, and/or dysphotopsia). All patients who met the indication criteria were given the option of surgery to replace with another IOL to improve contrast sensitivity, or follow-up without surgery. After sufficient informed consent, the treatment was chosen by the patient himself.

### Surgical technique

All the surgeries were performed by the same experienced surgeon (RT). The primary cataract surgery used a standard phacoemulsification technique under local anesthesia. A 2.4–3.0 mm clear corneal incision was made at the steepest corneal meridian, depending on the power and axis of the corneal astigmatism. Toric type IOLs were selected with 1.5 D or more for with-the-rule and 1.0 D or more for against-the-rule and oblique astigmatism. The corneal incision’s position and IOL axis were aligned using the VERION image guided system (Alcon, Fort Worth, Texas, USA).

The IOL exchange surgery used the same corneal incision of the previous cataract surgery. The corneal incision was opened, a viscoelastic material was injected, and the IOL was released from the capsular bag. The IOL optics were cut in half with scissors for easy explantation through the small wound and TECNIS Symfony^®^ was implanted in the capsular bag using an injector. No intraoperative complications were observed.

### Clinical evaluations

Patient demographics and clinical outcomes, including the visual acuity (VA), contrast sensitivity, subjective symptoms, time to IOL exchange, explanted IOL type, implanted IOL type, and postoperative spectacle independence, were investigated based on medical records. Waxy vision was defined as being equivalent to blurred vision, regardless of the sighting distance after spectacle correction.

The uncorrected and corrected distance VAs (UDVA and CDVA, respectively) were measured at 5 m before and after IOL exchange surgery. The uncorrected and distance-corrected near VAs (UNVA and DCNVA, respectively) were measured at 40 cm before IOL explantation. One month after implantation of TECNIS Symfony^®^, the uncorrected and distance-corrected intermediate VAs (UIVA and DCIVA, respectively) were measured at 70 cm. In some patients, the UNVA and DCNVA at 40 cm were also measured.

The contrast sensitivity was measured using the CSV-1000 instrument (Vector Vision, Fairfield, Connecticut, USA) under scotopic conditions with best spectacle correction. From the contrast sensitivity, the AULCSF was determined as described previously [12].

### Statistical analyses

All the statistical analyses were performed using R version 3.6.3 (The R Foundation for Statistical Computing, Vienna, Austria). The decimal VA values were converted to the logarithm of the minimum angle of resolution (logMAR) for analysis. The means ± standard deviations were used to describe the distributions of continuous variables, and percentages were used to describe the distributions of categorical variables. Univariate analysis was performed with the Wilcoxon signed-rank test. The tests of statistical significance were two-tailed, and p < 0.05 were considered statistically significant.

## Results

We analyzed the data for 29 eyes of 25 patients (10 males, 15 females). Table 1 shows the demographics of the study population before IOL exchange. The mean patient age was 62.5 ± 6.7 years (range: 49–75 years). The logMAR UDVA and CDVA were -0.07 ± 0.08 (-0.18–0.05) and -0.13 ± 0.06 (-0.18–0.00), respectively. Manifest spherical equivalent and cylinder values were 0.06 ± 0.34 D (-0.63–0.63 D) and 0.30 ± 0.30 D (0.00–0.75 D), respectively.

**Table 1:** Demographics of the patients before IOL exchange.

Demographic	Result
Sex (male/female)	10/15
Age (year)	62.5 ± 6.7
UDVA (logMAR)	-0.07 ± 0.08
CDVA (logMAR)	-0.13 ± 0.06
UNVA 40 cm (logMAR)	0.09 ± 0.16
DCNVA 40 cm (logMAR)	0.05 ± 0.13
Manifest spherical equivalent (D)	0.06 ± 0.34
Manifest cylinder (D)	0.30 ± 0.30
AULCSF	1.07 ± 0.12
Axial length (mm)	23.7 ± 1.6

UDVA = uncorrected distance visual acuity; CDVA = corrected distance visual acuity; UNVA = uncorrected near visual acuity; DCNVA = distance- corrected near visual acuity; AULCSF = area under the log contrast sensitivity function.

The time to the IOL exchange after the initial IOL implantation was 55.3 ± 50.4 days (range: 14–196 days). Explanted IOLs were TECNIS^®^ Multifocal ZLB00 (Johnson & Johnson Surgical Vision, Santa Ana, California, USA) in 23 eyes, AcrySof^®^ IQ ReSTOR^®^ +3.0 D (Alcon, Fort Worth, Texas, USA) in 2 eyes, and AcrySof^®^ IQ ReSTOR^®^ +3.0 D TORIC (Alcon, Fort Worth, Texas, USA) in 4 eyes. Diffractive bifocal IOLs were implanted in both eyes in 7 cases, of which monocular exchange was in 3 cases and binocular exchange was in 4 cases. If there was a difference in subjective symptoms between the eyes, the eye with more severe symptoms first underwent IOL exchange, and if there was no difference, the eye was IOL exchanged with the dominant eye.

Table 2 shows the visual and refractive outcomes 1 month after IOL exchange surgery. The logMAR UDVA and CDVA were 0.07 ± 0.28 (−0.18–0.70) and −0.14 ± 0.06 (−0.18–0.00), respectively. No statistically significant difference was seen in the logMAR CDVA before and after IOL exchange (p = 0.273). The AULCSF was significantly increased, from 1.07 ± 0.12 (0.80–1.27) preoperatively to 1.21 ± 0.12 (0.96–1.46) postoperatively (p < 0.001) (Fig 1). A significant increase in contrast sensitivity was observed at all 5 spatial frequencies after IOL exchange (Table 3).

**Fig 1:** Contrast sensitivity at 5 spatial frequencies before and after intraocular lens (IOL) exchange. IOL exchange induced a significant increase in contrast sensitivity at all spatial frequencies after surgery. Bar represents standard deviation.

**Table 2:** Visual and refractive outcomes after IOL exchange.

Demographic	Result
UDVA (logMAR)	0.07 ± 0.28
CDVA (logMAR)	-0.14 ± 0.06
UIVA 70 cm (logMAR)	-0.03 ± 0.08
DCIVA 70 cm (logMAR)	-0.04 ± 0.10
UNVA 40 cm (logMAR)	0.14 ± 0.15 *
DCNVA 40 cm (logMAR)	0.28 ± 0.15 *
Manifest spherical equivalent (D)	-0.36 ± 0.47
Manifest cylinder (D)	0.39 ± 0.34
AULCSF	1.21 ± 0.12

UDVA = uncorrected distance visual acuity; CDVA = corrected distance visual acuity; UIVA = uncorrected intermediate visual acuity; DCIVA = distance- corrected intermediate visual acuity; AULCSF = area under the log contrast sensitivity function.

*Analysis data of 21 eyes.

**Table 3:** Comparison of preoperative and postoperative the mean log contrast sensitivity.

Spatial Frequency	Preoperative	Postoperative	P Value
3 cpd	1.41 ± 0.16	1.57 ± 0.14	0.002
6 cpd	1.64 ± 0.15	1.78 ± 0.16	<0.001
12 cpd	1.23 ± 0.26	1.47 ± 0.28	<0.001
18 cpd	0.77 ± 0.26	0.99 ± 0.22	<0.001

cpd = cycles per degree.

The spectacle independence rate was 88.0% at the last visit. Three patients using spectacles were non-monovision binocular TECNIS Symfony^®^-implanted patients with the intended emmetropia or -1.0 D mild myopia targets. The purpose of using spectacles was for near vision in 2 cases and for distance vision in 1 case, and they were only used occasionally when necessary. As for subjective symptoms, disappearance of waxy vision was observed in 23 patients. Mild monocular waxy vision symptoms remained in 2 patients, but the symptoms were less than before IOL exchange surgery and spectacle independence was achieved, so they did not want any further intervention.

## Discussion

Even if the indications for multifocal IOL transplantation are carefully considered before surgery and good VA is obtained after surgery, some patients may not be satisfied with the surgical outcomes. In this study, patients who complained of waxy vision despite good UDVA after implantation of diffractive bifocal IOLs were exchanged for EDOF IOL and showed improvement in contrast sensitivity and subjective symptoms. Replacement with EDOF IOL, which provides comparable contrast sensitivity to that of monofocal IOL [10, 11], was considered one of the useful surgical options for cases of dissatisfaction with waxy vision after diffractive bifocal IOLs implantation.

Kamiya et al. [4] conducted a survey that included 50 eyes of multifocal IOL explantation in and reported that the most common visual complaint was waxy vision (29 eyes, 58%) and the most common reason for IOL explantation was decreased contrast sensitivity (18 eyes, 36%). Additionally, replacement surgery with monofocal IOL significantly increased the contrast sensitivity and improved patient satisfaction in the subgroup analysis of eyes whose contrast sensitivity was significantly decreased preoperatively. Diffractive bifocal IOLs tend to suppress the contrast sensitivity due to the optical characteristics dividing the focal point between far and near [1, 8–10]. Contrastingly, TECNIS Symfony^®^ is one of the EDOF IOLs that was able to suppress the decrease in the contrast sensitivity due to its proprietary diffractive echelette design and achromatic technology [10, 11, 13]. This can explain the difference in contrast sensitivity, owing to the difference in the structure of the IOLs, that was reflected in the results of this study.

Blurred vision is the main cause of dissatisfaction in patients with multifocal IOLs. Previous reports examining cases of dissatisfaction after implantation of multifocal IOLs reported that approximately 95% of the causes of dissatisfaction were blurred vision [5, 7]. Most of these cases improved with refractive surgery, spectacles, and YAG laser posterior capsulotomy, but some required replacement with monofocal IOL. IOL exchange is the last treatment and should be carefully considered and excluded from other possible factors in advance. Refractive error [4, 5, 7] and astigmatism of 1.0D or greater [14, 15] may affect visual function, but in this study the manifest spherical equivalent and cylinder values were within ±0.75D. Contrast sensitivity and near VA of the eyes with multifocal IOLs are susceptible to even mild posterior capsule opacification [16]. Shah et al. [17] reported that eyes implanted with multifocal IOLs required YAG laser capsulotomy on mean 8.8 months after surgery, which was earlier than that required in eyes implanted with monofocal IOLs. In this study, the period of IOL exchange was early (1.8 months), and symptoms were observed immediately after the initial cataract surgery in all cases; thus, it was considered that there was no effect of posterior capsule opacification.

There are concerns about the risk of complications when exchanging IOLs [4, 6, 18–20]. Regarding the complications during multifocal IOL exchange, Kamiya et al. [4] reported that the time to IOL exchange in 50 eyes was 7.9 months (3 days–40.5 months), 3 eyes (6%) required anterior vitrectomy, and 1 eye (2%) displayed partial zonular dehiscence. Galor et al. [6] reported that the mean time in 12 eyes was 13.6 months (2.1–18.9 months), 4 eyes required anterior vitrectomy, and 5 eyes displayed partial zonular dehiscence. In the current study, IOL exchange of 22 eyes was performed relatively early at 1.8 months (14 days–6.5 months), no intraoperative complications were observed, and IOL could be implanted in the capsular bag in all cases. Over time after cataract surgery, adhesion of the IOL to the capsular bag makes IOL explantation difficult. In addition, previous reports included cases after YAG laser capsulotomy, but in this study, YAG laser capsulotomy was not performed in consideration of the possibility of IOL exchange. The incidence of perioperative anterior vitrectomy in IOL exchange correlates with preoperative YAG laser capsulotomy [20]. IOL exchange should be considered by identifying the cause of dissatisfaction early before IOL adhesions, and YAG laser capsulotomy should be deferred as long as possible.

Hybrid monovision with monofocal IOL in the dominant eye and a multifocal IOL in the nondominant contralateral eye may reduce the waxy vision caused by bilateral multifocal IOL implantation [21, 22]. Several studies reported that EDOF IOL in the dominant eye and diffractive bifocal IOL in the nondominant contralateral eye may provide excellent good visual outcomes with minimal ocular symptoms [23, 24]. In this study, 2 of the 6 patients with bilateral implantation of diffractive bifocal IOLs, achieved improved waxy vision by exchanging only the dominant eye IOLs. If patients with bilateral diffractive bifocal IOL complain of waxy vision, it may be useful to first replace only the dominant eye with EDOF IOL.

The spectacle independence rate after multifocal IOL implantation averaged 80.1% in 63 studies [1], and that of EDOF IOL with micro-monovision was reported to be 84.0–88.6% [25, 26]. Conversely, monofocal IOLs were reported to be 17.2–25.8% [27–29]. In this study, the spectacle independence rate was 88.0%. The three patients using spectacles were non-monovision binocular EDOF IOL-implanted patients and used spectacles only occasionally. Patients undergoing cataract surgery with multifocal IOLs have high expectations for postoperative spectacle independence. The replacement with EDOF IOL, which can reduce the dependence on postoperative spectacles compared to monofocal IOL, is considered acceptable to patients.

Factors causing dissatisfaction after multifocal IOL implantation are not only restricted to waxy vision but also to poor VA and photic phenomena, and cases have been reported in which exchange monofocal IOLs were required [4–7]. Although less frequent than diffractive bifocal IOLs, photic phenomena, such as halos, glare, and starbursts, are also observed in EDOF IOL-implanted eyes, and some patients complain of severe symptoms [30]. Patients with poor VA, significantly decreased contrast, or severe photic phenomena should undergo monofocal IOL replacement.

There are several limitations of this study. First, this was a retrospective study; a randomized controlled study with exchanges to monofocal IOLs may provide further information confirming the validity of these results. Second, it is not possible to assess whether the results of this study are specific to the TECNIS Symfony^®^ or common to different types of EDOF IOLs, since there was no control group. Additionally, the number of patients analyzed was small, and the subjective symptoms were confirmed by interview, and a questionnaire survey on satisfaction was not conducted. However, since no patient wanted further surgical intervention after IOL exchange, we believe that patient satisfaction was obtained.

In conclusion, our study suggests that IOL exchange is a surgical option for dissatisfied patients with waxy vision in diffractive bifocal IOL-implanted eyes. Although monofocal IOLs are generally used as IOLs to be replaced, this study suggested that replacement with EDOF IOL is also effective. Further studies with more subjects using questionnaires on overall patient satisfaction, comparisons with replacement to monofocal IOLs, and verification of different types of EDOF IOLs are required to confirm these findings.

## Supporting information

S1 Table All relevant data in this manuscript. (XLSX)
